# LOXL2 Upregulation in Gliomas Drives Tumorigenicity by Activating Autophagy to Promote TMZ Resistance and Trigger EMT

**DOI:** 10.3389/fonc.2020.569584

**Published:** 2020-10-29

**Authors:** Qing Zhang, Lianhe Yang, Gefei Guan, Peng Cheng, Wen Cheng, Anhua Wu

**Affiliations:** ^1^Department of Neurosurgery, The First Hospital of China Medical University, Shenyang, China; ^2^Department of Pathology, First Affiliated Hospital and College of Basic Medical Sciences of China Medical University, Shenyang, China

**Keywords:** lysyl-oxidase-like-2, epithelial-to-mesenchymal transition, temozolomide, autophagy, glioma

## Abstract

Glioma is the most prevalent primary brain tumor in adults and has an extremely unfavorable prognosis. As a member of the lysyl oxidase (LOX) family, lysyl-oxidase-like-2 (LOXL2) is known to play different roles in different tumors. However, the role of LOXL2 in glioma has not yet been fully elucidated. In the present study, we detected that LOXL2 was considerably upregulated in glioma and that LOXL2 upregulation was evidently related to glioma WHO grade, malignant molecular subtypes, and poor prognosis in glioma patients. Additionally, we found that LOXL2 not only promoted glioma cells proliferation, migration, invasion, and induced the epithelial-to-mesenchymal transition (EMT) process, but also reduced the sensitivity of glioma cells to temozolomide (TMZ). Furthermore, we identified that LOXL2 reduced TMZ sensitivity and induced EMT in glioma *via* the activation of autophagy. Mechanistically, LOXL2 enhanced Atg7 expression by promoting the phosphorylation of Erk1/2, leading to the activation of autophagy and regulation of EMT process and TMZ sensitivity through autophagy. Our study describes an LOXL2-Erk1/2-Atg7 signaling axis that influences glioma EMT and chemosensitivity through autophagy; moreover, LOXL2 may serve as a promising therapeutic target in the treatment of glioma.

## Introduction

Glioma is the most prevalent form of primary intracranial tumor in adults (1). Even with aggressive surgery, radiation, and chemotherapy, compared with other tumors, the five-year survival rate of glioma patients is the most inferior (2). Moreover, survival time of patients with glioblastoma multiforme (GBM) averages a only 14 months after diagnosis (3).

As secreted amine oxidases, the main function of LOX family members is to covalently cross-link elastin and collagen in the extracellular matrix (ECM), which are indispensable to maintain the structural integrity of many tissues (4). LOXL2 is believed to perform an analogous function to LOX by promoting the cross-linking of collagen and elastin in the ECM. It has also been confirmed that LOXL2 can regulate signaling pathways inside or outside the cell (5). Disorders of LOXL2 have been related to a number of diseases, such as fibrosis (6) and heart disease (7). The expression and function of LOXL2 in tumor progression depends on tissue type. Although decreased expression level has been informed in ovarian tumors (8), LOXL2 is overexpressed and linked with unfavorable outcomes in patients with colon and esophageal tumors (9), squamous cell carcinoma in oral, head and neck, or laryngeal (10–12). In addition, over-expression of LOXL2 has been verified to promote tumor metastasis (13, 14). However, the function and specific mechanisms of LOXL2 in glioma have not been fully elucidated thus far.

TMZ is a first-line medicine used in the treatment of patients with glioma. The ultimate efficacy of TMZ varies according to intrinsic and acquired resistance, which greatly undermines its use in clinical treatment. Therefore, TMZ resistance is a primary handicap to the treatment of glioma, and research on TMZ resistance is vital to restore therapeutic efficacy and relieve the suffering of patients.

Autophagy is an extremely conservative mechanism of lysosome-mediated protein and organelle degradation that has an important effect on survival, differentiation, development, and homeostasis (15). In cancer, autophagy not only suppresses tumorigenesis *via* its quality control function, it also withstands microenvironmental stress and promotes malignant phenotype (16). In glioma, autophagy not only reduces TMZ sensitivity (17), it also modifies other processes including EMT, increasing the degree of malignancy (18). However, the specific regulatory mechanism of autophagy on TMZ sensitivity and EMT in gliomas has not been fully explained.

Here, we first explored the expression and prognostic efficacy of LOXL2 in The Cancer Genome Atlas (TCGA), Chinese Glioma Genome Atlas (CGGA), GSE16011 and the Repository for Molecular Brain Neoplasia Data (REMBRANDT), then detected its functions in tumorigenesis, EMT, and sensitivity to TMZ in glioma cells. The results suggested that high expression of LOXL2 is an important cause of glioma pathogenesis and TMZ resistance in glioma cells that might become a new target for glioma treatment.

## Materials and Methods

### Gene Expression Analysis Using Online Databases

Gene expression data and clinical characteristics (tumor grade, age at diagnosis, survival time, censored status, and treatment history) from TCGA for patients with GBM and low-grade glioma (LGG) were acquired from the cBioPortal for Cancer Genomics (http://www.cbioportal.org/datasets). Kaplan−Meier curves were developed *via* GraphPad Prism 7 (GraphPad Software Inc., San Diego, CA, USA), comparing overall survival rates between patients with and without the genetic alterations of interest. Survival differences were assessed by the log-rank test. Biospecimen and clinical data were collected and organized as introduced in TCGA publications (19). Progression-free survival data regarding GBM were obtained from Affymetrix arrays.

The CGGA database (http://www.cgga.org.cn) were also used in this study. Data from mRNAseq_693 were used for chemotherapy-related survival analyses. Other analyses were implemented using mRNAseq_325 data.

GSE16011 dataset were obtained through the Gene Expression Omnibus (GEO) database. Raw data were processed using the *affy* package, and the robust multi-array analysis (RMA) method was used for background correction and normalization. Biospecimen and clinical data from related research (20) were used as supplements.

The gene expression data and clinical information from REMBRANDT were acquired from the GlioVis portal (http://gliovis.bioinfo.cnio.es).

GSE43107 patient samples were collected in a Phase III randomized clinical trial, EORTC26951, that investigated adjuvant procarbazine, CCNU (lomustine), and vincristine (PCV) chemotherapy in anaplastic oligodendroglial tumors (21). A total of 140 patients out of the original 368 underwent expression profiling. Of these, 45 had profiling from HU133plus 2.0 arrays and 95 from exon arrays (HuEx_1.0_st arrays). Given the significant differences between these two platforms, we included samples only from exon arrays. Raw gene expression data and patient characteristics were obtained through the GEO database. Raw data were processed using the *Oligo* package and only the core probe set was analyzed for gene expression. The method of background correction and normalization is the same as that of GSE16011 data. mRNA expression was summarized with a BrainArray custom CDF file (22).

### Specimens and Patient Data

The protocol for our study was permitted by the Medical Ethics Committee of the First Affiliated Hospital of China Medical University. All patients involved in this study signed an informed consent agreement. Fifty-six glioma biospecimen were gathered from 2016 to 2018 in the First Hospital of China Medical University. **Supplementary Table 1** shows the clinicopathological information of these 56 samples. During the same period, an additional six samples were collected from people who had endured severe central nervous system trauma and underwent surgery immediately afterwards were used as a control group. These six patients were free of history of other central nervous system diseases. All 56 samples were subjected to qRT-PCR experiments, 12 of which and 1 non-tumor tissue were randomly selected for western blotting verification. All enrolled patients did not receive any other treatment before surgery.

### Cell Culture and Reagents

Normal human astrocyte (NHA) cell line and glioma cell lines, U373, U251, and U87 were obtained from the Chinese Academy of Sciences Cell Bank (Shanghai, China). T98 cells were acquired from the American Type Culture Collection (ATCC, Manassas, VA, USA). LN229 was handselled by Professor Tao Jiang (Department of Molecular Neuropathology, Beijing Neurosurgical Institute). All the cells were cultured as monolayer in Dulbecco’s Modified Eagle’s Medium (DMEM; Hyclone, Logan, UT, USA) supplemented with 10% fetal bovine serum (FBS), penicillin (100 U/ml), and streptomycin (100 U/ml) and incubated at 37°C with 5% carbon dioxide. Dimethyl sulfoxide (DMSO), chloroquine (CQ), 3-methyladenine(3-MA), and rapamycin were purchased from Sigma company (Sigma, St. Louis, MO, USA) and PD98059 was acquired from MedChemExpress (MedChemExpress, Monmouth Junction, NJ, USA).

### Quantitative Real-Time PCR

TRIzol Reagent (Invitrogen/Thermo Fisher Scientific, Waltham, MA, USA) was applied to extract the total RNA. The first-strand cDNA was synthesized *via* Prime-Script RT Master Mix (Takara Bio Inc., Shiga, Japan). SYBR Green Master Mix (TaKara, Japan) was applied to conduct qPCR detection (PCR LightCycler^®^ 480; Roche Diagnostics Ltd., Basel, Switzerland). Each sample was checked in triplicate. The specificity of the amplification was assessed by the dissolution curve. Relative mRNA expression levels were computed *via* the 2^-ΔΔCt^ formula. The following is the primer sequence of GAPDH and LOXL2:

GAPDH forward: 5’-GGAGCGAGATCCCTCCAAAAT-3’;

GAPDH reverse: 5’-GGCTGTTGTCATACTTCTCATGG-3’;

LOXL2 forward: 5’-GGCACCGTGTGCGATGACGA-3’;

LOXL2 reverse: 5’-GCTGCAAGGGTCGCCTCGTT-3’.

### Migration and Invasion Assays

Wound healing test was adopted to assess the migratory potential of cells. The ratio of wound closedown was detected at specified time points under a microscope and quantified *via* Image J (National Institutes of Health, Bethesda, Maryland, USA). Invasion potential was evaluated using collagen-coated Transwell assays (Corning, 8 µm; Corning, NY, USA). Serum free DMEM was supplemented to the upper wells and DMEM containing 10% FBS was supplemented to the lower wells. Cells invaded to the lower surface of the matrigel-coated filter in 20 h were counted.

### Western Blot Assays

Tissues or differently processed cells were collected and lysed *via* a protein extraction agent (Beyotime, Beijing, China). Total protein was quantified using the bicinchoninic acid (BCA) (Beyotime) method. In each lane, 25–50 μg protein per sample was loaded for sodium dodecyl sulfate-polyacrylamide gel electrophoresis (SDS-PAGE) and shifted onto PVDF membranes (0.45 μm, Millipore, NY, USA). After blocked by 5% skim milk solution for 1 h, the membranes were hatched with the indicated antibodies at 4°C for 16 h. The membranes were then hatched with the corresponding horseradish peroxidase-conjugated secondary antibodies at 20°C for 1 h. Immunoreactive proteins were visualized and quantified *via* a chemiluminescence reagent (Beyotime, Beijing, China) with a ChemiDoc™ Touch detection system (Bio-Rad Laboratories, Hercules, CA, USA) and Image J software. Detailed information of all antibodies is shown in **Supplementary Table 2**.

### Colony Formation, Cell Proliferation, and Cytotoxicity Assays

Cells were sown into 6-well plates (1,000 cells per well) and hatched for two weeks to test the ability of colony formation. Colonies containing more than 50 cells were counted.

Cell proliferation and cytotoxicity were checked *via* CellTiter 96^®^ AQueous One Solution Cell Proliferation Assay kits (Promega, Madison, WI, USA) for MTS assays. Cells were sown into five 96-well plates at 1,000 cells/100 μl per well and evaluated daily for 5 d. For cytotoxicity assays, 5,000 cells/100 μl were inoculated per well for three days. Cell viability was computed by the ratio of absorbance of each well at each time point to that of the control group (23).

### Transmission Electron Microscopy

Cells were first fixed in 2% glutaric acid and 1% osmium tetroxide in turn, then the cells were dehydrated and embedded in epoxy resin, and finally 50 nm slices were stained with lead citrate, and observed *via* a transmission electron microscope (H -7650, Hitachi, Japan).

### Apoptosis Assay

Apoptosis was checked using an Annexin V-PE/7-AAD double staining kit (BD Pharmingen Inc., San Diego, CA, USA) according to the manufacturer’s protocol. In short, harvested cells were cleaned by PBS and suspended in 1 × binding buffer. Aliquots of 10^5^ cells were stained with 5 μl of Annexin V/PE and 10 μl of 7ADD. Stained cells were detected *via* flow cytometry.

### RNA Interference, Plasmid Construction, and Lentiviruses

LOXL2, Erk1/2, and Atg7 were knocked down by specific small interfering RNAs (siRNAs) acquired from Sangon Biotech (Shanghai, China).The LOLX2 expression plasmid was obtained from GeneChem (Shanghai, China) with the corresponding empty vector (EV) as the control. Lipofectamine 3000 Reagent (Invitrogen, Carlsbad, CA, USA) was adopted for transfection of siRNAs, plasmid, or EV. Lentivirus carrying the LOXL2 siRNA sequence was obtained from Genechem. Puromycin (10 g/ml) was applied to screen out the stable transfected cells.

siRNAs used for the depletion of endogenous LOXL2, Erk1/2, and Atg7 had the following sequences:

LOXL2 siRNA sense, 5’-GGAGUUGCCUGCUCAGAAATT-3’;

antisense, 5’-UUUCUGAGCAGGCAACUCCTT-3’;

Erk1 siRNA sense, 5’-CCCUGACCCGUCUAAUAUAdTdT-3’;

antisense, 5’-UAUAUUAGACGGGUCAGGGdAdG-3’;

Erk2 siRNA sense, 5’-CAUGGUAGUCACUAACAUAdTdT-3’;

antisense, 5’-UAUGUUAGUGACUACCAUGdAdT-3’;

Atg7 siRNA sense, 5’-ATGATCCCTGTAACTTAGCCCA-3’;

antisense, 5’-CACGGAAGCAAACAACTTCAAC-3’.

### Tumor Xenograft Model

Six-week-old female athymic nude BALB/C mice were provided by Beijing Vital River Laboratory Animal Technology Company (Beijing, China) and fostered in laminar flow cabinets under specific pathogen-free (SPF) conditions in the Laboratory Animal Center of China Medical University. Animals used in this study were handled according to the China Medical University Animal Ethics Committee guidelines as agreed by the Animal Research Committee of China Medical University.

After the mice were anesthetized, their scalps were opened with a scalpel so that the skull was clearly displayed in the operation area. At a 3 mm depth from the skull surface, a 5 μl microsyringe containing a 3 μl cell suspension (5 × 10^5^ cells in PBS) was vertically injected into the brain 2 mm laterally and 2 mm anteriorly to the bregma. Finally, the mouse scalp skin was sutured to prevent infection. We assigned five mice to each group.

TMZ therapy was started a week after the operation. The mice were administered intraperitoneal injections of TMZ (5 mg/kg) or the same dose of DMSO. Drug were administered with a 5 days on/2 days off regimen, for two cycles. The entire brain of each mouse was incised in a coronal position from front to back. After staining with hematoxylin and eosin (H&E), the tumor location in each section was checked from anterior to posterior. The section with the largest tumor area was chosen to calculate tumor size. Tumor volume was calculated using the formula Volume = 1/2 mn^2^, where “m” represents the longest diameter and “n” stands for the shortest diameter.

### Statistical Analysis

In this study, GraphPad Prism version 6.0 (GraphPad Software, San Diego, CA, USA) and SPSS version 16.0 (SPSS Inc., Chicago, IL, USA) were applied for statistical analysis. One-way analysis of variance (ANOVA), two-tailed t test and log-rank test were applied to the corresponding conditions. Survival difference was determined by Kaplan−Meier analysis. Unless otherwise stated, p < 0.05 was believed statistically significant. Data are shown as the mean ± SEM or SD (3 or 5 experiments). *P < 0.05; **P < 0.01; ***P < 0.005, ****P < 0.001, ns: P ≥ 0.05.

## Results

### Gene Expression Profile Showed That LOXL2 Expression Was Linked to Glioma Grade and Prognosis

To survey the expression profiles of LOXL2 in gliomas, TCGA samples including 4 nontumor brain tissue samples and 664 glioma samples were analyzed. Of the 664 glioma samples, 246 (37.0%) were assorted as World Health Organization (WHO) grade II, 263 (39.6%) as grade III, and 155 (23.3%) as grade IV. LOXL2 expression was markedly more downregulated in WHO grade II glioma samples than in those graded III and IV (**Figure 1A**). An obvious divergence in LOXL2 expression levels was observed between tumors graded WHO III and IV (**Figure 1A**). These data indicated that there was a notable correlation between the level of LOXL2 expression and the grade of glioma. To further examine LOXL2 expression in gliomas across WHO grades, we conducted a similar analysis in CGGA and GSE16011 cohorts. The findings were consistent with those obtained in TCGA cohort (**Figures 1B, C**). Further analysis suggested that LOXL2 mRNA was downregulated in nontumor brain tissues compared to gliomas in TCGA dataset (**Figure 1A**). These findings suggested that increased LOXL2 mRNA expression was correlated with the genesis and progression of gliomas.

**Figure 1:** The expression characteristics of LOXL2 in the public database. LOXL2 levels were checked in different grades **(A)**, subtypes **(D)**, and isocitrate dehydrogenase (IDH) mutation statuses **(G)** in The Cancer Genome Atlas (TCGA) cohort. LOXL2 expression levels assessed in different grades **(B)**, subtypes **(E)**, and IDH mutation statuses **(H)** in the Chinese Glioma Genome Atlas (CGGA) cohort. LOXL2 expression levels assessed in different grades **(C)**, subtypes **(F)**, and IDH mutation statuses **(I)** in the GSE16011 cohort. Kaplan-Meier ananlysis examined the relationship between LOXL2 and overall survival of patients with all gliomas **(J)**, LGG **(K)**, and GBM **(L)** in TCGA. *P < 0.05; **P < 0.01; ***P < 0.005.

Using the public databases mentioned above, Kaplan−Meier analysis found that high expression levels of LOXL2 in glioma, LGG, and GBM predicts poor overall survival (**Figure 1J–L**, **Supplementary Figures 1A–H**), consistent with the results of previous clinical case studies (24). All these data indicated that the expression of LOXL2 was not only correlated with the occurrence and development of glioma, but also linked with the outcomes of glioma patients.

### LOXL2 Was a Signature of Glioma Subtype

TCGA divides GBM into four molecular subtypes based on gene expression, they are classical, mesenchymal, neural, and proneural subtypes (25). Independent of grade, the presence of isocitrate dehydrogenase (IDH) mutations in gliomas confers appreciably better progression-free survival than that associated with IDH wild-type, regardless of treatment (26). To assess whether LOXL2 expression could help distinguish glioma subtypes, we used TCGA, CGGA, and GSE16011 cohorts. We found that the expression level of LOXL2 in the mesenchymal subtype was much higher than that in the other three subtypes in all three datasets (**Figures 1D–F**). In addition, the expression levels of LOXL2 in IDH wild type were also significantly higher than those in the IDH mutant type in the three datasets (**Figures 1G–I**). The above results indicated that the expression levels of LOXL2 were closely related to the malignant subtype of glioma, and might affect glioma’s response to therapy.

### LOXL2 Upregulation in Glioma Tissues and Glioma Cell Lines and LOXL2 as a Predictor of TMZ Response in Glioma

This study assessed 6 normal brain tissue samples, 18 grade II specimens, 20 grade III specimens, and 18 grade IV specimens to determine LOXL2 expression in tumor and nontumor. In the samples, we found that LOXL2 mRNA levels were notably higher in gliomas than in nontumor brain tissue (**Figures 2A, B**). Additionally, LOXL2 expression significantly increased with higher WHO glioma grades (**Figures 2A, B**). Protein level analysis on randomly selected samples yielded consistent results (**Figure 2C**). In addition, regardless of protein level or mRNA level, the expression level of LOXL2 in glioma cell lines was much higher than that of NHA (**Figures 2D, E**).

**Figure 2:** LOXL2 expression verified in glioma samples and cell lines and LOXL2 was a predictor of response to temozolomide (TMZ) in glioma. **(A, B)** LOXL2 mRNA expression were analyzed by qRT-PCR in 56 glioma samples and 6 normal brain tissues. **(C)** Western blots showed that LOXL2 expression was significantly increased in glioma samples compared to non-tumor tissues. GAPDH was used as a control. LOXL2 mRNA **(D)** and protein **(E)** expression levels checked by qRT-PCR and western blots in glioma cells (U373, U87, U251, LN229, and T98) and normal human astrocyte (NHA). **(F, G)** KM curves for GSE43107 on the basis of median LOXL2 expression. Samples were grouped according to treatment modality (IR alone and IR + alkylating chemotherapy). **(H, I)** Survival curves of The Cancer Genome Atlas (TCGA) HG-U133A platform data based on median LOXL2 expression. Patients with glioblastoma multiforme (GBM) were grouped according to treatment modality (IR alone and TMZ chemotherapy with or without IR). **(J, K)** Survival curves of Chinese Glioma Genome Atlas (CGGA) (mRNAseq_693) data on the basis of median LOXL2 expression. Samples receiving chemotherapy were categorized according to diagnosis [low-grade glioma (LGG) and GBM]. **(L, M)** Progression-free survival (PFS) curves in LGG and GBM of TCGA on the basis of median LOXL2 expression. *P < 0.05; **P < 0.01; ***P < 0.005.

To understand whether LOXL2 was involved in alkylation damage, we looked at three independent expression databases. One was the European Organization for Research and Treatment of Cancer (EORTC) study 26951 (21). The EORTC study was conducted prior to the routine use of TMZ, and LOXL2 expression did not affect the overall survival rate of patients receiving only IR treatment (**Figure 2F**). But for patients who received both alkylating chemotherapy and IR treatment, the prognosis of patients with low expression level of LOXL2 is significantly better than that of patients with high LOXL2 expression level (**Figure 2G**). In TCGA database (HG-U133A), LOXL2 expression level did not affect outcome among GBM patients treated with IR alone (**Figure 2H**). For GBM patients receiving TMZ treatment, patients with low LOXL2 expression levels had a more favorable prognosis than patients with high expression levels (**Figure 2I**). To validate these results for LOXL2, we examined another glioma expression dataset, CGGA. Among patients who received chemotherapy, those whose tumors exhibited low LOXL2 expression levels had a much better prognosis for both LGG (**Figure 2J**) and GBM (**Figure 2K**). The LOXL2 expression level identified in TCGA database were also inversely related to progression-free survival (PFS) (**Figures 2L, M**). Altogether, the above data not only further verified the relationship between LOXL2 expression and WHO grade of glioma, but also indicated that LOXL2 expression affects response of glioma to the TMZ treatment.

### Knockdown of LOXL2 Inhibited Glioma Cells Proliferation, Migration, Invasion, and EMT

We explored the function of LOXL2 in the occurrence and development of glioma by silencing LOXL2 expression with siRNA in glioma cells. The LOXL2 expression level was significantly decreased by siRNA compared with negative-control cells (**Supplementary Figures 2A, C**). Colony formation and MTS assay results suggested that the knockdown of LOXL2 obviously suppressed the proliferation of U87 and U251 cells (**Figures 3A, B**). Wound healing tests and Transwell assays found that LOXL2 silencing notably restrained migration (**Figure 3C**) and invasion (**Figure 3D**) ability of glioma cells. To investigate the mechanism by which LOXL2 regulated glioma cell proliferation and motility, we assessed the expression of Cyclin D1, MMP-2, and MMP-9. Their expression levels obviously declined after LOXL2 knockdown (**Figure 3E**).

**Figure 3:** LOXL2 silencing restrained glioma cells amplification, motility, and epithelial-to-mesenchymal transition (EMT) *in vitro*. U87 **(A)** and U251 **(B)** cell amplification slowed after LOXL2 knockdown, measured *via* colony formation and MTS assays. **(C, D)** Glioma cells motility decreased following LOXL2 knockdown; scale bar = 100 µm. **(E)** Western blotting showed that LOXL2 silencing inhibited the expression of cell cycle regulatory protein cyclin D1 and invasion-related proteins MMP-2 and MMP-9. **(F)** Western blotting showed the regulation of EMT-related proteins after LOXL2 knockdown. **(G)** Immunofluorescence analysis verified that LOXL2 silencing inhibited the expression of vimentin and N-cadherin; scale bar = 100 µm. **P < 0.01; ***P < 0.005.

EMT is a biological process regulated by many proteins, which allows tumor cells to gain strong invasive ability, thereby promoting tumor progression and metastasis (27). To survey whether the effect of LOXL2 on glioma motility was related to EMT, we checked the expression of EMT-related markers. Following a reduction in LOXL2 expression, the expression levels of Vimentin, N-cadherin, ZEB1, β-catenin, Claudin-1, and SLUG were downregulated; in contrast, the expression level of E-cadherin was upregulated (**Figure 3F**). The results of immunofluorescence assays for Vimentin and N-cadherin expression were consistent with those obtained *via* western blotting (**Figure 3G**). This finding suggested that the regulation of glioma motility by LOXL2 may be related to EMT.

### LOXL2 Overexpression Promoted Glioma Cell Proliferation, Invasion, Migration, and EMT

To further evaluate the function of LOXL2 on the tumorigenesis and progression of glioma, we assessed the role of LOXL2 overexpression in glioma cells and confirmed the results obtained *via* western blotting and qPCR (**Supplementary Figures 2B, D**). Colony formation and MTS assays suggested that LOXL2 overexpression promoted the proliferation of glioma cells (**Supplementary Figures 3A, B**). In addition, the migration and invasion potential of glioma cells were also strengthened in LOXL2 overexpressed glioma cells (**Supplementary Figures 3C, D**). After LOXL2 overexpression, the expression levels of the cell cycle and motility-related markers, Cyclin D1, MMP-2, and MMP-9 also increased significantly (**Supplementary Figure 3E**).

Overexpression and silencing of LOXL2 yielded opposite results regarding the expression of EMT-related proteins (**Supplementary Figures 2F, G**). These data suggest that LOXL2 improved the invasion ability of glioma cells by promoting EMT. The positive correlation between the expression of LOXL2 and EMT markers (Vimentin, N-Cadherin, Slug, Claudin-1) in TCGA and CGGA datasets further confirmed this result (**Supplementary Figures 4–A**).

### LOXL2 Mediated Glioma Cell Resistance to Temozolomide

TMZ is widely used in the clinical treatment of glioma. Considering that LOXL2 had a strong predictive ability for the prognosis of glioma patients receiving TMZ treatment, we speculated that LOXL2 might regulate the sensitivity of glioma cells to TMZ. To verify this conjecture, we treated U87 and U251 cells with different concentrations of TMZ. Cells that overexpressed LOXL2 had higher viability than those in the control group after TMZ treatment; LOXL2 silencing conferred hypersensitivity to TMZ in both cell lines compared with control group (**Figures 4A, B**, **Supplementary Figures 5A, B**). The IC50 for TMZ of glioma cells in different transfection groups further confirmed these results (**Supplementary Figures 5–C**). We also observed that the expression levels of LOXL2 in U87 and U251 cells were dose- and time-dependent on TMZ (**Figures 4C, D**). To investigate whether regulation of the sensitivity to TMZ brought on by LOXL2 in glioma cells was affected by apoptosis, the function of LOXL2 on glioma cell apoptosis was checked by flow cytometry. LOXL2 had no effect on cell apoptosis (**Figures 4E, F**) or expression of caspase-3 and cleaved caspase-3 (**Figures 4G, H**). Together, these results suggested that LOXL2 mediated glioma cell resistance to TMZ.

**Figure 4:** LOXL2 promotes temozolomide (TMZ) tolerance in glioma cells. **(A, B)** Cell viabilities with LOXL2 knockdown and overexpression in U87 **(A)** and U251 **(B)** upon treatment with indicated TMZ doses for 72 h. **(C)** Western blotting of LOXL2 expression with TMZ (200 µM) exposure for indicated time. **(D)** Western blotting of LOXL2 expression with TMZ exposure at indicated concentrations for 72 h. **(E, F)** Flow cytometry analysis found that LOXL2 had no effect on the apoptosis of glioma cells. **(G)** Overexpression of LOXL2 in glioma cells regulated the expression of apoptosis-related proteins caspase-3, cleaved caspase-3, and autophagy-related proteins Beclin-1, P62, LC3-I, and LC3-II. **(H)** LOXL2 silencing in glioma cells regulated the expression of apoptosis-related proteins caspase-3, cleaved caspase-3, and autophagy-related proteins Beclin-1, P62, LC3-I, and LC3-II. *P < 0.05; **P < 0.01; ***P < 0.005, ns: P ≥ 0.05.

### Autophagy Was Responsible for LOXL2-Induced Temozolomide Resistance and LOXL2-Induced EMT in Glioma Cells

There are many mechanisms that regulate the tolerance of glioma cells to TMZ, including O6-methylguanine-DNA methyltransferase (MGMT), protective autophagy, and stemness of glioma cells (28). However, there is no notable correlation between the expression levels of LOXL2 and MGMT, nor the expression levels of LOX2 and glioma stem cell markers (OLIG2 and CD133) (**Supplementary Figure 6**). Autophagy is an extremely conservative catabolic process that can provide cells with certain nutrients to better adapt to the changes in the environment (29). It is one of the important reasons for tumor resistance to radiotherapy and chemotherapy (30, 31). In addition, studies have confirmed that autophagy can promote the occurrence of EMT in glioma cells (32, 33). Thus, we explored whether LOXL2 regulated autophagy in glioma cells.

Western blotting showed that the expression of LC3-II and Beclin-1 were elevated and the expression of P62 was decreased in LOXL2-transfected glioma cells (**Figure 4G**). The opposite effect was observed in cells that silenced LOXL2 (**Figure 4H**). The intensity of the autophagy was evaluated by the expression levels of LC3-I and LC3-II with or without rapamycin (Rapa) or 3-methyladenine (3-MA). Western blotting revealed that the expression of LC3-II decreased after 3-MA treatment; compared to the combination of EV and 3-MA, the combination of LOXL2-overexpression and 3-MA increased the expression of LC3-II (**Figure 5A**). Treatment of LOXL2-knockdown cells with Rapa reversed the decreased expression of LC3-II with si-LOXL2 alone (**Figure 5B**). Using fluorescence microscopy, we discovered that the number of autophagosome paralleled the expression of LOXL2 (**Figure 5C**). Additionally, TME scan also found that overexpression of LOXL2 promoted autophagy, while silencing LOXL2 inhibited autophagy in glioma cells (**Figure 5D**). These results suggested that LOXL2 was capable of activating autophagy. In glioma tumor tissues, we also detected that the expression of LOXL2 was related to the intensity of autophagy (**Supplementary Figure 7**).

**Figure 5:** LOXL2 induces temozolomide (TMZ) resistance and epithelial-to-mesenchymal transition (EMT) *via* activating autophagy in glioma cells. **(A)** LC3-I and LC3-II expression changed with LOXL2 overexpression and 3-MA (10 mM, 48 h) treatment. **(B)** LC3-I and LC3-II expression levels variated with LOXL2 knockdown and rapamycin (Rapa) (50 nM, 48 h) treatment. **(C)** Glioma cells with transduced stubRFP-LC3 with LOXL2 overexpression or silencing, the stubRFP-LC3 punctuate localization was analyzed by fluorescence microscopy; scale bar = 40 µm. **(D)** Autophagy was evaluated in U87 and U251 cells under different transfections using TEM. Red arrows, autophagic structure; scale bar =1 µm. **(E)** Viability of control cells or LOXL2-overexpressing cells with or without CQ (5 µM, 72 h) with indicated TMZ doses. **(F)** Invasion ability of glioma cells treated with EV, LOXL2, LOXL2+CQ (5 µM, 48 h); scale bar = 100 µm. **(G)** Expression of EMT-related proteins in glioma cells treated with EV, LOXL2 and LOXL2+CQ (5 µM, 48 h). *P < 0.05; **P < 0.01, ***P < 0.005, ****P < 0.001, ns: P ≥ 0.05.

Consistent with previous findings (31), glioma cells treated with TMZ showed increased autophagy intensity (**Supplementary Figures 8A, B**). To explore whether LOXL2 regulated tolerance to TMZ by activating autophagy, we studied the regulation of LOXL2 on TMZ tolerance using the autophagy inhibitor CQ. We found that CQ reversed TMZ tolerance resulting from LOXL2 overexpression at a CQ concentration that did not affect cell viability (**Supplementary Figure 8C** and **Figure 5E**).

We further explored whether the promotional effect of LOXL2 on EMT is produced by autophagy. We found that CQ can reverse the promotion of LOXL2 on glioma cell migration (**Supplementary Figures 9A, B**) and invasion (**Figure 5F**) and can inhibit the expression of EMT-related markers (**Figure 5G**) caused by LOXL2 overexpression. The regulatory effect of 3-MA on LOXL2 overexpression cells in TMZ sensitivity and EMT was similar to that of CQ (**Supplementary Figure 10**). However, in LOXL2 silenced cells, 3-MA or CQ had no significant effect on the TMZ sensitivity and migration and invasion ability of the cells. There was also no difference in the expression of EMT-related proteins and LC3 (**Supplementary Figure 11**). Collectively, these results suggested that LOXL2-induced TMZ resistance and LOXL2-induced EMT may, at least in part, have been due to the activation of autophagy.

### LOXL2 Regulated Autophagy by Controlling Atg7 Expression

To clarify the specific mechanism of LOXL2 stimulating autophagy in glioma cells, we assessed the expression of five key autophagy regulators (Atg7, Atg16L1, Atg12, Atg5, and Atg3) in LOXL2-overexpressing and -knockdown cells. Only the expression of Atg7 varied with the expression of LOXL2 (**Figure 6A**); in other words, overexpression of LOXL2 can promote the expression of Atg7, while knockout of LOXL2 can inhibit the expression of Atg7. According to the TCGA, CGGA, and GSE16011 databases, the expression level of Atg7 increased with the increasing of LOXL2 expression level (**Supplementary Figures 12A–C**). To verify this finding, we designed an Atg7-specific siRNA to knockdown expression of Atg7 in LOXL2-overexpressing glioma cells (**Supplementary Figure 13A**). We found that silencing Atg7 could reverse the expression of LC3-II caused by the overexpression of LOXL2 (**Figure 6B**). In addition to western blotting, stubRFP-LC3 staining and TEM indicated that Atg7 knockout inhibited autophagy caused by overexpression of LOXL2 (**Figures 6C, D**). This suggests that the regulation of autophagy by LOXL2 depends on its regulation of Atg7 expression.

**Figure 6:** LOXL2 affects autophagy by regulating Atg7 expression. **(A)** LOXL2 regulated Atg7 expression but not Atg5, Atg3, Atg12, or Atg16L1. **(B)** Expression of Atg7, EMT-related markers, LC3-I and LC3-II in differently transfected glioma cells. **(C)** Immunofluorescence of stubRFP-LC3 punctuate localization in glioma cells with EV, LOXL2, and LOXL2 + si-Atg7 treatment; scale bar = 40 µm **(D)** Autophagy evaluated in glioma cells with EV, LOXL2, and LOXL2 + si-Atg7 treatment using TEM. Red arrows, autophagic structure; scale bar = 1 µm. **(E)** Immunofluorescence determined the Vimentin and N-cadherin expression in differently transfected glioma cells; scale bar = 100 µm. **(F, G)** Wound healing **(F)** and Transwell assays **(G)** in glioma cells to compare migration and invasion potential with EV, LOXL2, and LOXL2 + si-ATG7 treatment; scale bar = 100 µm. **(H)** Cell viabilities of control cells or LOXL2-overexpressing cells with or without Atg7-specific siRNA and indicated TMZ doses. *P < 0.05; **P < 0.01, ns: P ≥ 0.05.

Furthermore, when endogenous Atg7 was silenced, the expression levels of EMT-related markers resulting from LOXL2 overexpression were partially reversed (**Figures 6B, E**). Silencing Atg7 also significantly inhibited the migration and invasion potential of glioma cells, even with LOXL2 overexpression (**Figures 6F, G**). Compared with LOXL2 overexpression alone, the sensitivity of glioma cells to TMZ increased with LOXL2 overexpression and Atg7 knockdown (**Figure 6H**).

Since Atg7 has a powerful regulatory effect on autophagy (34), many studies have used Atg7 knockout as a way to inhibit autophagy (35). Knocking down Atg7 here to suppress autophagy not only reversed LOXL2’s regulation of EMT in glioma cells, but also inhibited LOXL2’s regulation of glioma cell tolerance to TMZ. The above results indicated that LOXL2 promoted TMZ tolerance and EMT of glioma cells by promoting autophagy.

### LOXL2 Regulated Atg7 Expression by Promoting the Phosphorylation of Erk1/2

We further investigated the mechanism by which LOXL2 regulated Atg7. We discovered that LOXL2 regulated the phosphorylation of Erk1/2 (**Supplementary Figure 13B** and **Figure 7A**). In addition, using the Erk1/2 inhibitor PD98059 and Erk1/2 specific si-RNA (**Supplementary Figure 13C**), we found that LOXL2 affected Atg7 expression by regulating the phosphorylation of Erk1/2, which further affected the expression of LC3-II (**Figure 7A**). Using fluorescence microscopy, we detected a decrease in the number of stubRFP-LC3 puncta in LOXL2-upregulated cells with PD98059 or Erk1/2-specific siRNA treatment compared with LOXL2-overexpression alone (**Figure 7B**). This suggests that LOXL2 can promote Erk1/2 phosphorylation to facilitate the expression of ATG7, thus promoting autophagy.

**Figure 7:** LOXL2 regulated Atg7 expression by promoting Erk1/2 phosphorylation. **(A)** Protein levels of Erk1/2, p-Erk1/2, Atg7, epithelial-to-mesenchymal transition (EMT)-related markers, LC3-I, and LC3-II in differently transfected glioma cells. **(B)** Immunofluorescence of stubRFP-LC3 punctuate localization in U87 and U251 cells with EV, LOXL2, LOXL2 + PD98059, and LOXL2 + si-Erk1/2 treatment; scale bar = 40 µm **(C)** Immunofluorescence was used to assess Vimentin and N-cadherin expression in glioma cells under different transduction conditions; scale bar = 100 µm. **(D)** Wound healing and **(E)** Transwell assays of glioma cells for comparison of cell migration and invasion with EV, LOXL2, LOXL2 + PD98059, and LOXL2 + si-Erk1/2 treatment; scale bar = 100 µm. **(F)** Viability of glioma cells with EV, LOXL2, LOXL2 + PD98059, and LOXL2 + si-Erk1/2 with indicated TMZ doses. *P < 0.05; **P < 0.01, ns: P ≥ 0.05.

In addition, knockout of Erk1/2 or the use of Erk1/2 inhibitor PD98059 can also reverse the changes in EMT related protein expression caused by overexpression of LOXL2 (**Figures 7A, C**). The migration and invasion abilities of glioma cells were also inhibited in LOXL2-overexpressing cells treated with PD98059 or Erk1/2-specific si-RNA (**Figures 7D, E**). Sensitivity to TMZ also increased with this treatment (**Figure 7F**). These results indicated that LOXL2 activated autophagy by promoting Erk1/2 phosphorylation to increase the expression of Atg7, thereby triggering EMT and promoting TMZ tolerance in glioma cells.

### LOXL2 Silencing Increased the Sensitivity of Glioma Cells to TMZ *In Vivo*

Orthotopic xenograft models were adopted to further confirm the function of LOXL2 on the tumorigenesis of glioma and the sensitivity of glioma cells to TMZ. The overall survival of nude mice was tracked after intracranial injection of U87 cells with or without stable silencing of LOXL2 and with or without intraperitoneal administration of TMZ. The results showed that the stable silencing of LOXL2 or TMZ treatment alone slightly prolonged the overall survival of the nude mice and slowed the growth of tumors (**Figures 8A–C**). The combination treatment of TMZ with stable silencing of LOXL2 significantly prolonged overall survival and inhibited the growth of tumors (**Figures 8A–C**). In addition, the median survival time of mice receiving both TMZ treatment and inoculation with LOXL2 stably silenced U87 cells (37.5 days) was obviously prolonged compared to that of the control group (21 days), TMZ treatment alone (26.5 days) or LOXL2 stable silenced alone (26.5 days) groups. These results demonstrated that LOXL2 was important for glioma tumorigenesis and TMZ resistance.

**Figure 8:** LOXL2 affects the occurrence of glioma and temozolomide (TMZ) tolerance *in vivo*. **(A)** HE staining images of glioma sections obtained from mice bearing intracranial xenografts from U87 cells (transduced with either si-NC or si-LOXL2 containing lentivirus) with or without TMZ treatment. Scale bar = 1 mm. **(B)** Tumor size in different treatment groups. **(C)** KM analysis of mice with orthotopically transplanted U87 cells and different treatments (n = 5). *P < 0.05; **P < 0.01, ***P < 0.005.

## Discussion

In summary, our data described the potential mechanism by which LOXL2 regulated autophagy in glioma. LOXL2 is a pivotal factor in EMT in various cancers (36, 37). LOXL2 overexpression promotes the formation of the collagen fiber network in the ECM, which is considered to be one of the direct causes of liver fibrosis and cirrhosis (6), pulmonary fibrosis (38), and the occurrence of some tumors (39). However, the biological role of LOXL2 and its specific mechanism in glioma have not been fully elucidated

Our research shows that the LOXL2 expression levels were obviously correlated with the grade of glioma, and were negatively associated with the overall survival of glioma patients in the four public databases. The former was further conformed using qRT-PCR and western blotting on glioma samples of different grades and glioma cell lines, indicating that LOXL2 plays a functional role in the pathogenesis of glioma. Further analysis revealed that TMZ treatment significantly prolonged the overall survival of glioma patients with low LOXL2 expression.

Next, we evaluated the function of LOXL2 in glioma cells. LOXL2 silencing significantly inhibited cell multiplication, migration, and invasion. LOXL2 silencing suppressed the EMT process and increased TMZ sensitivity in glioma cell lines. Overexpression and silencing of LXOL2 yielded the opposite results.

Further investigation showed that LOXL2 might affect glioma cells through the regulation of Atg7 expression by promoting Erk1/2 phosphorylation. Over 30 autophagy regulators have been detected in yeast and most of which are highly conserved in mammals (40). Among them, Atg7 regulates autophagy by regulating LC3 and ATG5/12-related ubiquitination reactions (41). Atg7 is important for the occurrence and development of many tumors and tumor chemoradiotherapy resistance by regulating autophagy (42). Erk1/2 has also been confirmed to be important in the occurrence and progression of many tumors (43). Similar to LOXL2 knockdown, PD98059 or Erk1/2-specific siRNA inhibited the effects of LOXL2 on the regulation of Atg7 expression, which further affected the process of EMT and sensitivity to TMZ by inhibiting glioma cell autophagy. As far as we know, this is the first report to provide detailed evidence that LOXL2 activates autophagy to promote EMT and increase TMZ tolerance in glioma.

However, the detailed mechanism of the relationship between LOXL2 expression and histological grade remains unclear. Hypoxia plays an important role in both chemoradiotherapy resistance and unfavorable prognosis (44). Hypoxia-inducible-factor-1 (HIF-1-alpha) can upregulate LOXL2 expression, as LOXL2 has a hypoxia response element (HRE) in its promoter region (45). This may be one reason why LOXL2 expression is associated with histological grade. Besides, it has been reported that hydrogen peroxide (H2O2) is the product of LOXL2 catalytic reaction (46, 47); moreover, H_2_O_2_ activates Erk1/2 (48). This may explain why LOXL2 can activate Erk1/2, but the specific mechanism requires further study.

The specific mechanism of autophagy’s regulation of EMT requires further study. Studies in hepatocellular carcinoma have reported that autophagy activated the cAMP/PKA/CREB or TGFβ/Smad3 signaling pathway to promote EMT (49, 50). In lung adenocarcinoma, the co-culture of mesenchymal stem cells and lung adenocarcinoma cells can promote the activation of autophagy in lung adenocarcinoma cells, thereby up-regulating the expression of Snail and promoting the occurrence of EMT in lung adenocarcinoma cells (51). These indicate that the regulation of EMT by autophagy is a complex process involving a variety of signal pathways and biological processes and that further efforts are needed to fully reveal it. As for the role of autophagy in chemotherapy response in cancer, different studies have opposite conclusions (52–55). The activation of Erk1/2 pathway was not only confirmed to be closely related to the occurrence and development of many tumors, but also promoted autophagy (56). In our study, LOXL2 can not only predict the prognosis of patients receiving TMZ treatment, but also regulates the Atg7-Erk1/2 signaling pathway to promote autophagy of glioma cells, and increases the tolerance of glioma cells to TMZ. These results illuminate why LOXL2 can promote glioma chemotherapy resistance through autophagy.

In conclusion, our research confirmed that LOXL2 promoted the occurrence and progression of glioma and reduced the response of glioma cells to chemotherapy. It also manifested that a combination of LOXL2 inhibitor or antibody and TMZ may offer greater efficacy for the clinical treatment of patients with glioma. Moreover, it would be of interest in the field of oncology to assess whether our conclusions can be generalized to the therapy of other tumors.

## Data Availability Statement

The cohorts used in this study can be acquired through http://www.cgga.org.cn/ (CGGA), http://www.cbioportal.org/datasets (TCGA), https://www.ncbi.nlm.nih.gov/geo/ (GEO), http://gliovis.bioinfo.cnio.es/ (REMBRANDT). Further enquiries can be directed to the corresponding author.

## Ethics Statement

The studies involving human participants were reviewed and approved by The Medical Ethics Committee of the First Hospital of China Medical University. The patients/participants provided their written informed consent to participate in this study. The animal study was reviewed and approved by The Institutional Animal Research Committee of China Medical University.

## Author Contributions

The experimental design was completed by QZ and AW, and the experimental operation, data collection, and analysis were conducted by QZ. QZ and AW wrote the manuscript, and all authors checked and corrected it. All authors contributed to the article and approved the submitted version.

## Funding

Our study was funded by grants from the National Natural Science Foundation of China (grant numbers: 81172409, 81472360, and 81872054), and Liaoning Science and Technology Plan Projects (grant number: 2011225034).

## Conflict of Interest

The authors declare that the research was conducted in the absence of any commercial or financial relationships that could be construed as a potential conflict of interest.
